# Assessment of the Potential Adverse Events Related to Ribavirin-Interferon Combination for Novel Coronavirus Therapy

**DOI:** 10.1155/2020/1391583

**Published:** 2020-09-24

**Authors:** Wenya Shan, Dongsheng Hong, Jieqiang Zhu, Qingwei Zhao

**Affiliations:** ^1^Department of Clinical Pharmacy, The First Affiliated Hospital of Zhejiang University, 310003, China; ^2^Zhejiang University of Technology, 310003, China; ^3^Zhejiang Provincial Key Laboratory for Drug Evaluation and Clinical Research, 310003, China

## Abstract

**Purpose:**

We aimed to analyze and evaluate the safety signals of ribavirin-interferon combination through data mining of the US Food and Drug Administration Adverse Event Reporting System (FAERS), so as to provide reference for the rationale use of these agents in the management of relevant toxicities emerging in patients with novel coronavirus pneumonia (COVID-19).

**Methods:**

Reports to the FAERS from 1 January 2004 to 8 March 2020 were analyzed. The proportion of report ratio (PRR), reporting odds ratio (ROR), and Bayesian confidence interval progressive neural network (BCPNN) method were used to detect the safety signals.

**Results:**

A total of 55 safety signals were detected from the top 250 adverse event reactions in 2200 reports, but 19 signals were not included in the drug labels. All the detected adverse event reactions were associated with 13 System Organ Classes (SOC), such as gastrointestinal, blood and lymph, hepatobiliary, endocrine, and various nervous systems. The most frequent adverse events were analyzed, and the results showed that females were more likely to suffer from anemia, vomiting, neutropenia, diarrhea, and insomnia.

**Conclusion:**

The ADE (adverse drug event) signal detection based on FAERS is helpful to clarify the potential adverse events related to ribavirin-interferon combination for novel coronavirus therapy; clinicians should pay attention to the adverse reactions of gastrointestinal and blood systems, closely monitor the fluctuations of the platelet count, and carry out necessary mental health interventions to avoid serious adverse events.

## 1. Introduction

Since December 2019, the novel coronavirus pneumonia (COVID-19) has exploded in China and spread to many countries and regions around the world. At present, there is no clinically effective antiviral drug for COVID 19; according to the antiviral treatment recommended by China, ribavirin is suggested to be used in combination with interferon or lopinavir/ritonavir.

Ribavirin (RBV) is a purine nucleoside analogue with broad-spectrum antiviral activity, which can be used in combination with interferon (IFN) for the treatment of chronic hepatitis C [1], and was also an empirical treatment regimen during the outbreak of the Middle East respiratory syndrome coronavirus (MERS-CoV) [2]. The drug labels list the possible adverse drug events (ADEs), but less attention has been paid to the potential adverse events related to ribavirin-interferon combination, mainly including lower respiratory tract infection, suicide attempt, gastrointestinal ulcer, cerebral hemorrhage, mental disorder, and hallucinations. Studies have confirmed that ribavirin-interferon combination can lead to arteriosclerosis [3] and even cause heart enlargement in patients to develop into dilated cardiomyopathy [4]. However, all these ADEs are not listed in the drug labels, due to the delay of the update of the labels and the complexity of united medication. Ribavirin-interferon combination was recommended for the treatment of COVID-19 [5], but there was less information on the ADEs. A spontaneous reporting system is an important data source for monitoring ADEs in the world, and the FDA established the US Food and Drug Administration Adverse Event Reporting System (FAERS) database to support postmarketing surveillance programs. The real-world data can provide information to help clinicians weigh the risks and benefits of these agents. Therefore, we aimed to analyze and evaluate the safety signals of ribavirin-interferon combination through data mining of the FAERS, in order to assess the potential adverse events related to the combination for novel coronavirus therapy.

## 2. Methods

### 2.1. Data Source

The FDA publishes FAERS files every quarter, and each quarterly file package contains the following seven data files: demographic and administrative information, drug information, adverse drug reaction information, patient outcome information, drug therapy start dates and end dates, information on report sources, and indications for use/diagnosis [6]. The adverse events are coded using the Preferred Terms (PTs) from the Medical Dictionary for Regulatory Activities (MedDRA).

In this study, a research AE analysis tool was used to extract adverse events from the FAERS database. Searches were performed using both the generic and brand names of ribavirin and interferon, and the reports were included when ribavirin and interferon were both suspected to be the primary agent. The top 250 adverse events were retrieved from the FAERS database which covered the period from 1 January 2004 to 8 March 2020.

### 2.2. Data Mining Algorithm

A spontaneous reporting system is an important data source for monitoring adverse drug reactions in the world and finding the signals of adverse drug reactions after marketing. To identify drug-associated adverse events as signals, a disproportionality analysis is regarded as a fundamental tool of analytic methods, which compares the proportion of occurring adverse events between the study drug and all other drugs [7]. While disproportionality analysis includes the frequency and Bayesian methods, no “gold standard” is available, and each of the above methods has its own characteristics [8]. Both the proportional reporting ratio (PRR) [9] and reporting odds ratio (ROR) [10] are frequency methods. They are easy for calculation and can lead to a more sensitive output than Bayesian approaches. However, frequency measures are extremely sensitive to small fluctuations in the number of reports. Results are not always credible in the event of small numbers in cells a, b, c, and d in a two-by-two frequency table. The Bayesian confidence propagation neural network (BCPNN) [11] is always applicable and large numbers of calculations can be made efficiently, but it is relatively nontransparent for people unfamiliar with Bayesian statistics. No one algorithm is universally better than others. In order to reduce the bias of a single algorithm, PRR, ROR, and BCPNN were used to detect the signals. The combination of three signal mining methods can improve the sensitivity and specificity of adverse event signal detection, reducing the false-positive rate to ensure the reliability of signal detection results. These algorithms extract decision rules for evaluating associations between drugs and adverse events from a two-by-two frequency table of counts that involve the presence or absence of the study drug and the particular event occurring in case reports (see Table 1).

For the PRR and ROR, a signal is detected if the lower bound of the 95% two-sided confidence interval (CI) exceeds 1.0. Using the BCPNN, IC‐2SD > 0 results in a signal, and the algorithm is shown in Equation (1). In this study, adverse events were listed as drug-associated, when all three indices met the aforementioned criteria. The higher the scores of PRR, ROR, and BCPNN, the stronger the association between drugs and adverse events.

(1) $$\begin{array}{c} \alpha_{1}=\beta_{1}=1,\alpha =\beta =2,\gamma_{11}=1,C=a+b+c+d,C_{x}=a+b,C_{y}=a+c,C_{xy}=a,\gamma =\gamma_{11}\frac{\left(C+\alpha \right)\left(C+\beta \right)}{\left(C_{x}+\alpha_{1}\right)\left(C_{y}+\beta_{1}\right)},E\left(\text{IC}\right)=\log_{2}\frac{\left(C_{xy}+\gamma_{11}\right)\left(C+\alpha \right)\left(C+\beta \right)}{\left(C+\gamma \right)\left(C_{x}+\alpha_{1}\right)\left(C_{y}+\beta_{1}\right)},\\ V\left(\text{IC}\right)=\frac{1}{{\left(\ln2\right)}^{2}}\left\{\left(\frac{C-C_{xy}+\gamma -\gamma_{11}}{\left(C+\gamma_{11}\right)\left(1+C+\gamma \right)}\right)+\left(\frac{C-C_{x}+\alpha -\alpha_{1}}{\left(C_{x}+\alpha_{1}\right)\left(1+C+\alpha \right)}\right)+\left(\frac{C-C_{y}+\beta +\beta_{1}}{\left(C_{y}+\beta_{1}\right)\left(1+C+\beta \right)}\right)\right\},\\ \text{IC}-2\text{SD}=E\left(\text{IC}\right)-2\sqrt{V\left(\text{IC}\right)}. \end{array}$$

## 3. Results

### 3.1. Ribavirin and Interferon-Associated Adverse Events

During the study period, a total of 2200 adverse event reports were reported with ribavirin and interferon as the first suspected drugs. Demographic characteristics of patients and composition of serious adverse events are shown in Table 2. A total of 827 reports were from medical staff, accounting for 37.59% of all reports. In terms of gender composition, 1128 reports were linked to males, which accounted for 51.27% of all reports, and the age was concentrated at 45-64 years. Serious adverse events after combined use accounted for 44.60%, of which the most frequently reported cases were hospitalization or prolonged hospitalization.

### 3.2. Signal Detections for RBV and IFN

A total of 55 positive signals were detected from the top 250 adverse event reactions in 2200 reports and described according to their System Organ Class (SOC), as defined in MedDRA. All the detected adverse event reactions were associated with 13 SOC, such as gastrointestinal, blood and lymph, hepatobiliary, endocrine, and various nervous systems (see Table 3). We counted the reports of each adverse event; the most frequent adverse events displayed according to SOC were gastrointestinal (426 reports, 19.56%), blood and lymphatic (360 reports, 16.35%), psychiatric (311 reports, 14.28%), medical examination (287 reports, 13.18%), and skin and subcutaneous tissues (286 reports, 13.13%) (see Figure 1).

In order to identify gender-specific differences in adverse events, the most frequent adverse events were analyzed by ROR. ROR > 1 indicates that females are more likely to have adverse reactions, and ROR < 1 indicates that males are more likely to have adverse reactions [12]. The results showed that females were more likely to suffer from anemia (ROR = 1.18), vomiting (ROR = 2.75), neutropenia (ROR = 1.97), diarrhea (ROR = 1.99), and insomnia (ROR = 1.40) than males (see Table 4).

According to the results, 19 signals were not included in the drug labels, which accounted for 34.55% of all safety signals, including ascites, splenomegaly, hemoptysis, and rectal bleeding. The list contains designated medical events (DME) containing medical conditions that are inherently serious and often medicine-related. In order to highlight the clinical relevance of the signals, we verified whether these PTs are listed in the DME provided by the European Medicines Agency (EMA). The results showed that hepatic failure (PPR = 4.96, ROR = 4.97, and IC‐2SD = 2.14) and hemoptysis (PPR = 2.63, ROR = 2.63, IC‐2SD = 1.17) were on the DME list.

## 4. Discussion

Previous research has shown that anemia, neutropenia, mood swings, and adverse reactions of the skin system were the most common adverse events in patients during the treatment of ribavirin-interferon combination [13–15]. In our research, anemia (256 reports, PRR = 12.45, ROR = 12.48, and IC‐2SD = 3.42), depression (149 reports, PRR = 5.32, ROR = 5.32, and IC‐2SD = 2.29), and rash (173 reports, PRR = 4.22, ROR = 4.22, and IC‐2SD = 1.96) were the signals that have the higher number of reports and PRR, ROR, and IC values in each system. The FDA adverse event database is mainly from patients with hepatitis, and the results of signal screening were consistent with the adverse reactions reported in the literature. The safety signal screening based on the FDA adverse event database indicates the potential ADEs related to ribavirin-interferon combination and can also provide a reference for novel coronavirus therapy.

According to the results, during the treatment of ribavirin-interferon combination, the most commonly reported adverse events were in the gastrointestinal system, mainly manifested as vomiting, diarrhea, abdominal distention, and other discomfort. Gastrointestinal adverse events will result in a loss of appetite and poor sleep quality, and even drug stoppage if things get worse. This will limit the use of antiviral drugs and affect the therapeutic effect of patients. Thus, how to reduce the gastrointestinal adverse events of patients with COVID-19 may be the focus of clinical attention. Health education can be carried out among patients by clinicians, so that patients can know the disease and drugs correctly. When patients realize that gastrointestinal reaction is a normal phenomenon, their uneasiness will be reduced. For patients with gastrointestinal discomfort, clinicians should provide timely symptomatic treatment, adjust the diet structure of patients, and reduce the stimulating food.

Ribavirin-interferon combination can also lead to blood and lymphatic system diseases and abnormal medical examination indicators. It has been proven that patients often suffer from anemia, thrombocytopenia, neutropenia, and other symptoms during the combined treatment [13, 14]. When ribavirin and interferon are coadministered in patients with COVID-19, close monitoring of the hemoglobin level is recommended. For patients with anemia, dose reduction is needed if there is an unknown reason for the decline of hemoglobin; ADEs should be identified. In a multicenter trial [16], one patient stopped treatment at the 42nd week of treatment due to the decrease of platelet to 45000/mm^3^. In another study [17], a case of death due to combined treatment was reported. At the start of treatment, the patient already had a rather low platelet count; the platelet further drops after the combined treatment and finally leads to death. Dosages were reduced according to the drug labels, but further dose reductions might be needed for this patient. This suggests that the abnormality of the medical examination index may cause serious adverse reactions and even death. For patients with a low blood cell count at the start of treatment, clinicians should reduce the dosages according to the drug labels and adjust the dose according to the situation of patients during the treatment to avoid serious adverse events.

Depression was a signal with a higher number of reports and PRR, ROR, and IC values in the nervous system. At present, studies have confirmed that patients undergoing treatment of ribavirin-interferon combination will increase the risk of diseases such as depression and anxiety [17, 18]. In the face of an outbreak, patients with COVID-19 may be lonely, anxious, and have insomnia and are more likely not to cooperate with the treatment due to fear of the disease. Clinicians need to objectively communicate with patients about the changes of disease and epidemic situation and encourage patients to cooperate with the treatment. In order to reduce the occurrence of adverse events and protect the mental health of patients, the involvement of a psychiatrist may be necessary. At the same time, this study analyzed the gender-specific differences of the 10 adverse events with the highest number of reports. Female patients may be more prone to mood swings, which may cause insomnia, vomiting, and other diseases.

According to the signal detection results, 19 signals were not listed in the drug labels, and they may be considered as unexpected. The biggest limitation of this approach is confounding by indication and failed to highlight the clinical relevance of the signals. For instance, ascites and splenomegaly are likely to be disease-related complications (HCV, with cirrhosis). Hepatic events are likely to be related to the underlying hepatic damage, but patients may also receive other hepatotoxic drugs. Hepatic failure and hemoptysis are the only two signals that are listed in the DME, which are inherently serious and often medicine-related. Although they are not listed in the drug labels, they indicate the possible adverse events in the treatment of ribavirin-interferon combination. A prospective multicenter study in Thailand [17] showed that a patient with HCV and HIV had severe hemoptysis after treatment with ribavirin-interferon combination and was consistent with our signal detection results. ADEs cannot be easily detected in studies conducted before the drug reaches the market; new adverse reports may appear after the drug is marketed, while the update of the drug label is lagging behind. Previous studies have shown ADEs that are not listed in the drug labels of ribavirin and interferon, such as aortosclerosis [3], dilated cardiomyopathy [4], leprosy [19], and glycosylated hemoglobin 1Ac reduction [20]. According to the results, clinicians should also pay attention to the adverse reactions of hepatic failure and hemoptysis. Especially for novel coronavirus-infected patients, adverse reactions may accelerate the progression of the disease and cause fatal risks.

In this study, signal detection is based on the spontaneous reporting database, which has some shortcomings such as missing reports and repeated reports. This study only focused on the adverse events of ribavirin-interferon combination, but did not take into account the basic diseases and other combined medications of patients. It is quite impossible to identify which patient is prescribed these drugs and for what reason. Also, we do not have information regarding how long patients were on one of the drugs prior to starting on combination therapy. The positive signals detected in this study only indicate that there is a statistical correlation between the drug and adverse events, and the clear causal correlation needs to be confirmed by further research.

## 5. Conclusions

Based on the FDA adverse event database, 55 positive signals were detected in this study. The most frequent adverse events displayed according to SOC were gastrointestinal system diseases, blood and lymphatic system diseases, psychiatric diseases, medical examination, and skin and subcutaneous tissue diseases. During the treatment of ribavirin-interferon combination, patients may have adverse reactions in the gastrointestinal and blood system, and pharmaceutical care should be strengthened to avoid serious adverse events. Hepatic failure and hemoptysis were the positive signals that are not listed in the drug labels but in the DME list. They were considered inherently serious and often medicine-related.

The signal detection and analysis by using the database of a spontaneous reporting system can warn of adverse events that may occur in the practical treatment of ribavirin and interferon. In the special environment of a new epidemic situation, it can provide reference for rationale use of these agents in the management of relevant toxicities emerging in patients with COVID-19.

## Figures and Tables

**Figure 1:** Number of adverse event reports associated with each SOC.

**Table 1:** Two-by-two frequency table.

	Adverse event of interest	All other adverse events	Total
Drug of interest	*a*	*b*	*a* + *b*
All other drugs	*c*	*d*	*c* + *d*
Total	*a* + *c*	*b* + *d*	*a* + *b* + *c* + *d*

**Table 2:** Demographic characteristics of patients and composition of serious adverse events.

Variables	Reports	Percentage
*Occupation*		
Physician	827	37.59%
Pharmacist	47	2.14%
Other health professional	563	25.59%
Lawyer	7	0.32%
Consumer or nonhealth professional	655	29.77%
Unknown	101	4.59%
*Gender*		
Male	1128	51.27%
Female	863	39.23%
Unknown	209	9.50%
*Age (y)*		
<18	22	1.00%
18-44	300	13.64%
45-64	872	39.77%
65-74	157	7.14%
≥75	11	0.50%
Unknown	835	37.95%
*Seriousness*		
Death	143	6.50%
Hospitalization	657	29.86%
Congenital anomalies	4	0.18%
Disabling	74	3.36%
Life threatening	103	4.68%

**Table 3:** All the detected adverse events displayed according to SOC and PT.

PT	Reports	PRR (95% CI)	ROR (95% CI)	IC (IC-2SD)	Listed in the drug labels
*Blood and lymphatic system disorders*					
Anemia	256	12.45 (11.09, 13.98)	12.48 (11.68, 13.34)	3.42 (3.22)	Yes
Neutropenia	87	7.40 (6.03, 9.10)	7.41 (6.65, 8.27)	2.74 (2.42)	Yes
Splenomegaly	9	6.48 (3.38, 12.45)	6.49 (4.65, 9.07)	2.06 (1.15)	No
Aplastic anemia	8	13.65 (6.83, 27.29)	13.68 (9.60, 19.51)	2.50 (1.54)	Yes
*Endocrine disorders*					
Hypothyroidism	31	9.36 (6.60, 13.28)	9.37 (7.82, 11.24)	2.88 (2.36)	Yes
Thyroid disorder	22	9.03 (5.95, 13.69)	9.04 (7.30, 11.20)	2.73 (2.12)	Yes
Hyperthyroidism	18	11.61 (7.33, 18.41)	11.64 (9.18, 14.75)	2.89 (2.36)	Yes
*Eye disorders*					
Visual acuity reduced	23	4.27 (2.84, 6.42)	4.28 (3.47, 5.27)	1.90 (1.30)	Yes
Retinal exudates	13	95.68 (55.36, 165.36)	97.48 (73.62, 129.09)	3.62 (2.85)	Yes
Vogt-Koyanagi-Harada syndrome	9	355.71 (180.91, 699.39)	382.31 (270.42, 540.51)	3.29 (2.37)	Yes
*Gastrointestinal disorders*					
Vomiting	107	2.04 (1.70, 2.45)	2.04 (1.85, 2.25)	0.98 (0.69)	Yes
Diarrhea	85	1.30 (1.05, 1.60)	1.30 (1.16, 1.45)	0.36 (0.03)	Yes
Abdominal pain	39	1.47 (1.08, 2.01)	1.47 (1.25, 1.73)	0.53 (0.07)	Yes
Ascites	31	8.55 (6.03, 12.14)	8.57 (7.15, 10.27)	2.78 (2.26)	No
Abdominal distension	26	2.23 (1.52, 3.27)	2.23 (1.83, 2.72)	1.08 (0.52)	Yes
Proctalgia	22	29.82 (19.65, 45.25)	29.99 (24.19, 37.17)	3.72 (3.11)	No
Hemorrhoids	22	8.95 (5.90, 13.56)	8.96 (7.23, 11.10)	2.72 (2.12)	No
Pancreatitis acute	21	7.34 (4.79, 11.23)	7.35 (5.90, 9.15)	2.50 (1.88)	Yes
Rectal hemorrhage	19	3.47 (2.22, 5.44)	3.47 (2.76, 4.38)	1.62 (0.97)	No
Mouth ulceration	14	6.10 (3.62, 10.28)	6.10 (4.67, 7.98)	2.18 (1.43)	Yes
Anorectal discomfort	13	16.62 (9.66, 28.60)	16.67 (12.62, 22.03)	2.97 (2.19)	No
Anal pruritus	10	24.09 (12.96, 44.78)	24.20 (17.61, 33.25)	2.96 (2.08)	No
Tooth loss	9	6.58 (3.43, 12.63)	6.59 (4.71, 9.20)	2.07 (1.16)	No
Irritable bowel syndrome	8	3.96 (1.98, 7.91)	3.96 (2.78, 5.65)	1.57 (0.61)	No
*General disorders and administration site conditions*					
Oedema peripheral	29	1.69 (1.18, 2.43)	1.69 (1.40, 2.04)	0.72 (0.18)	Yes
*Hepatobiliary disorders*					
Hepatic cirrhosis	56	27.84 (21.48, 36.08)	27.98 (24.43, 32.05)	4.22 (3.83)	No
Hepatic failure	34	4.96 (3.55, 6.93)	4.97 (4.18, 5.90)	2.14 (1.64)	No
Hepatic fibrosis	23	40.15 (26.69, 60.38)	40.46 (32.78, 49.93)	3.93 (3.33)	No
Hepatic function abnormal	15	3.47 (2.09, 5.75)	3.47 (2.68, 4.50)	1.58 (0.85)	Yes
Hepatotoxicity	9	4.27 (2.22, 8.20)	4.27 (3.06, 5.97)	1.68 (0.77)	Yes
Cholestatic hepatitis	9	11.83 (6.16, 22.73)	11.86 (8.49, 16.57)	2.50 (1.59)	No
*Investigations*					
Platelet count decreased	80	7.29 (5.88, 9.04)	7.30 (6.51, 8.18)	2.72 (2.38)	Yes
White blood cell count decreased	79	7.29 (5.87, 9.05)	7.30 (6.51, 8.19)	2.71 (2.38)	Yes
Hemoglobin decreased	72	5.91 (4.71, 7.42)	5.92 (5.25, 6.67)	2.43 (2.08)	Yes
Red blood cell count decreased	25	7.07 (4.79, 10.45)	7.08 (5.79, 8.66)	2.51 (1.94)	Yes
Blood creatinine increased	19	2.40 (1.53, 3.75)	2.40 (1.90, 3.02)	1.16 (0.51)	No
Haematocrit decreased	12	4.15 (2.36, 7.30)	4.15 (3.11, 5.55)	1.74 (0.93)	No
*Metabolism and nutrition disorders*					
Dehydration	42	2.55 (1.89, 3.44)	2.55 (2.18, 2.98)	1.28 (0.84)	Yes
Diabetes mellitus	30	3.15 (2.20, 4.49)	3.15 (2.62, 3.78)	1.54 (1.02)	Yes
Lactic acidosis	10	3.18 (1.71, 5.91)	3.18 (2.32, 4.37)	1.41 (0.53)	No
*Nervous system disorders*					
Loss of consciousness	28	1.77 (1.22, 2.56)	1.77 (1.46, 2.14)	0.78 (0.23)	Yes
Dysgeusia	21	2.18 (1.42, 3.34)	2.18 (1.75, 2.71)	1.04 (0.42)	Yes
Cerebral infarction	18	4.72 (2.98, 7.48)	4.72 (3.73, 5.98)	1.97 (1.31)	Yes
Hepatic encephalopathy	15	9.65 (5.82, 15.98)	9.66 (7.46, 12.53)	2.64 (1.91)	No
Facial palsy	11	23.63 (13.09, 42.67)	23.74 (17.53, 32.14)	3.03 (2.19)	No
*Psychiatric disorders*					
Depression	149	5.32 (4.55, 6.21)	5.32 (4.89, 5.79)	2.29 (2.04)	Yes
Insomnia	81	2.52 (2.04, 3.12)	2.52 (2.25, 2.83)	1.28 (0.95)	Yes
Anorexia	35	13.00 (9.36, 18.07)	13.03 (10.99, 15.46)	3.27 (2.78)	Yes
Suicidal ideation	30	2.61 (1.83, 3.72)	2.61 (2.17, 3.14)	1.30 (0.77)	Yes
Psychotic disorder	16	3.95 (2.42, 6.43)	3.95 (3.07, 5.08)	1.74 (1.04)	Yes
*Renal and urinary disorders*					
Renal impairment	18	2.16 (1.36, 3.42)	2.16 (1.70, 2.73)	1.02 (0.35)	Yes
*Respiratory, thoracic, and mediastinal disorders*					
Interstitial lung disease	13	2.32 (1.35, 3.99)	2.32 (1.76, 3.07)	1.08 (0.3)	Yes
Hemoptysis	9	2.63 (1.37, 5.04)	2.63 (1.88, 3.67)	1.17 (0.26)	No
*Skin and subcutaneous tissue disorders*					
Rash	173	4.22 (3.66, 4.87)	4.22 (3.90, 4.57)	1.96 (1.73)	Yes
Pruritus	113	3.35 (2.80, 4.01)	3.35 (3.04, 3.69)	1.66 (1.38)	Yes

**Table 4:** Gender differences in adverse event reactions.

SOC/PT	Reports	ROR (95% CI)
Anemia	256	1.18 (1.03, 1.35)
Rash	173	0.88 (0.76, 1.01)
Depression	149	1.04 (0.87, 1.24)
Pruritus	113	0.80 (0.65, 0.97)
Vomiting	107	2.75 (2.21, 3.42)
Neutropenia	87	1.97 (1.54, 2.50)
Diarrhea	85	1.99 (1.57, 2.53)
Insomnia	81	1.40 (1.10, 1.76)
Platelet count decreased	80	0.91 (0.72, 1.15)
White blood cell count decreased	79	0.83 (0.65, 1.05)

## Data Availability

All experimental data used in this study are available from the corresponding author upon request.
